The article "Tlr5 deficiency exacerbates lupus-like disease in the MRL/lpr mouse model" was retracted in 2024. Reasons: unreliable results or conclusions; concerns about the data; concerns about the images.

# *Tlr5* deficiency exacerbates lupus-like disease in the MRL/*lpr* mouse model

**DOI:** 10.3389/fimmu.2024.1359534

**Published:** 2024-01-30

**Authors:** Razan M. Alajoleen, David N. Oakland, Rana Estaleen, Aida Shakeri, Ran Lu, Michael Appiah, Sha Sun, Jonathan Neumann, Shimako Kawauchi, Thomas E. Cecere, Ryan P. McMillan, Christopher M. Reilly, Xin M. Luo

**Affiliations:** ^1^ Department of Biomedical Sciences and Pathobiology, Virginia-Maryland College of Veterinary Medicine, Virginia Polytechnic Institute and State University, Blacksburg, VA, United States; ^2^ Graduate Program of Translational Biology, Medicine, and Health, Virginia Polytechnic Institute and State University, Roanoke, VA, United States; ^3^ Department of Biological Sciences, College of Science, Virginia Polytechnic Institute and State University, Blacksburg, VA, United States; ^4^ Department of Developmental and Cell Biology, University of California, Irvine, Irvine, CA, United States; ^5^ Transgenic Mouse Facility, University of California, Irvine, Irvine, CA, United States; ^6^ Department of Human Nutrition, Foods and Exercise, Virginia Polytechnic Institute and State University, Blacksburg, VA, United States; ^7^ Department of Biomedical Sciences, Edward Via College of Osteopathic Medicine, Blacksburg, VA, United States

**Keywords:** lupus, TLR5, glomerulonephritis, lymphoproliferation, gut microbiota

## Abstract

**Introduction:**

Leaky gut has been linked to autoimmune disorders including lupus. We previously reported upregulation of anti-flagellin antibodies in the blood of lupus patients and lupus-prone mice, which led to our hypothesis that a leaky gut drives lupus through bacterial flagellin-mediated activation of toll-like receptor 5 (TLR5).

**Methods:**

We created MRL/*lpr* mice with global *Tlr5* deletion through CRISPR/Cas9 and investigated lupus-like disease in these mice.

**Result:**

Contrary to our hypothesis that the deletion of *Tlr5* would attenuate lupus, our results showed exacerbation of lupus with *Tlr5* deficiency in female MRL/*lpr* mice. Remarkably higher levels of proteinuria were observed in *Tlr5* ^-/-^ MRL/*lpr* mice suggesting aggravated glomerulonephritis. Histopathological analysis confirmed this result, and *Tlr5* deletion significantly increased the deposition of IgG and complement C3 in the glomeruli. In addition, *Tlr5* deficiency significantly increased renal infiltration of Th17 and activated cDC1 cells. Splenomegaly and lymphadenopathy were also aggravated in Tlr5^-/-^ MRL/*lpr* mice suggesting impact on lymphoproliferation. In the spleen, significant decreased frequencies of regulatory lymphocytes and increased germinal centers were observed with *Tlr5* deletion. Notably, *Tlr5* deficiency did not change host metabolism or the existing leaky gut; however, it significantly reshaped the fecal microbiota.

**Conclusion:**

Global deletion of *Tlr5* exacerbates lupus-like disease in MRL/*lpr* mice. Future studies will elucidate the underlying mechanisms by which *Tlr5* deficiency modulates host-microbiota interactions to exacerbate lupus.

## 1 Introduction

Systemic lupus erythematosus (SLE) is a complex autoimmune disorder characterized by a cascade of pathological events, such as the production of autoantigen-autoantibody immune complexes (ICs), the recruitment of autoreactive or inflammatory T cells, and the abnormal production of pro-inflammatory cytokines (1, 2). These immunological dysregulations conclude in severe inflammation and deposition of ICs in various peripheral tissues, resulting in organ damage that can affect the kidneys, lungs, joints, heart and brain, among other organs (1). Leaky gut has gained increasing attention as a potential contributor to the pathogenesis of autoimmune diseases, including SLE (3). A leaky gut referred to as increased intestinal permeability involves the disruption of the intestinal barrier, allowing for the passage of luminal antigens, toxins, and microbial components into the bloodstream (4). The gastrointestinal tract, beyond its primary role in digestion and nutrient absorption, serves as a critical interface between the external environment and the host immune system (5). The gut mucosa houses a vast community of microorganisms collectively known as the gut microbiota. These microbes play a crucial role in maintaining immune homeostasis and influencing systemic immune responses (5).

Flagellin, a protein component of bacterial flagella, has been hypothesized as a potential trigger of immune dysregulation in autoimmune diseases (6) including rheumatoid arthritis, SLE, and systemic sclerosis (7–9). An increased level of anti-flagellin IgG antibodies has also been linked to Crohn’s disease (10). Flagellin is recognized by Toll-like receptor 5 (TLR5), an innate immune receptor that plays a pivotal role in detecting bacterial infections to initiate an inflammatory response (11). Aberrant activation of TLR5 signaling, potentially driven by exposure to flagellin, has been implicated in the pathogenesis of SLE and its associated complications (12). The precise mechanisms underlying the development and progression of SLE are still under investigation, but recent research has shed light on the role of TLR5 signaling in this context. Dysregulated TLR5 signaling can lead to an overactive immune response, including the production of pro-inflammatory cytokines and the generation of autoantibodies against self-antigens (13, 14). It has also been suggested that TLR5 signaling may influence the balance of gut microbiota, affecting the intestinal homeostasis (15). Changes in the gut microbiota can, in turn, influence the immune system and potentially contribute to the autoimmune processes observed in SLE (16). Notably, we have recently shown that the levels of anti-flagellin antibodies are significantly upregulated in the blood of SLE patients and lupus-prone MRL/*lpr* mice (17). This has led to our hypothesis that bacterial flagellin-mediated activation of TLR5 would trigger SLE-like autoimmunity in lupus-prone MRL/*lpr* mice. To provide a comprehensive exploration of the intricate relationship between a leaky gut, flagellin-TLR5 signaling, and their potential impact on the development and progression of disease in SLE, we have assessed the development of autoimmune disease in our newly generated *Tlr5*-deficient lupus-prone MRL/*lpr* mice.

## 2 Materials and methods

### 2.1 Generation of *Tlr5* ^-/-^ MRL/*lpr* mice

Lupus-prone MRL/*lpr* mice (MRL/Mp-*Fas^lpr/lpr^*, stock number 000485) were purchased from The Jackson Laboratory (Bar Harbor, ME). Generation of *Tlr5*-null mice on MRL/*lpr* background was conducted by Transgenic Mouse Facility at University of California, Irvine, where we designed to directly modify the *Tlr5* gene in MRL/*lpr* zygotes, using CRISPR-CAS9 approach to save time and effort of intensive backcrossing. Four Alt-R CRISPR RNAs (TMF1931 – 5’- CAG AGA GCT AAT GTC TTC TG -3’, TMF1932 – 5’- CAC AGA AGA CAT TAG CTC TC -3’, TMF1933 – 5’- AAG GAC CCC CAG CGG CTG TG -3’, TMF1934 – 5’- GC TTT ATC CGC ACA GCC GCT -3’), and tracrRNA plus CAS9 protein (HiFi Cas9 nuclease V3, Integrated DNA Technologies, or IDT, Coralville, IA) as a ribonucleoprotein was electroporated into MRL/*lpr* mice to generate double stranded DNA breaks at the upstream and downstream of coding sequence of *Tlr5* (exon3 and exon4 in *Tlr5-203* transcript-ENSMUST00000193687.7). G0 founder mice were screened by PCR to identify animals having a deletion allele of *Tlr5* produced by removal of DNA in the vicinity of the CAS9 cut sites followed by non-homologous end joining repair. G0 animals containing a prospective deletion allele were backcrossed with MRL/*lpr* mice and N1F1 heterozygous mice were sequenced to determine the mutant allele. The *Tlr5*-null allele (*Tlr5* ^-/-^) has a deletion of 3493 bp of contiguous DNA from nucleotide position 182,799,888 to 182,803,380 on Chromosome 1. (Nucleotide position from mouse genome refers to build GRCm39, Ensembl release 110.) The deletion begins 112 nucleotides upstream of the translation initiation ATG codon in exon 3 and ends 61 nucleotides downstream of the translation STOP codon in exon 4. (CCACCACAGAAgacattagctctct.…tttatccgcacAGCCGCTGGGGGTCC: where the uppercase sequence is retained and the lowercase sequence is deleted.) Oligonucleotides for PCR-based genotyping were purchased from IDT (Coralville, IA). *Tlr5-null* genotyping was performed using primer sets, using a common forward primer and allele specific reverse primers to amplify both *Tlr5* wildtype allele and *Tlr5* null allele (Common Forward 5′- TATGGGGCCATTCTTCCTTGAA -3′; *Tlr5*-wildtype (Int3)-Rev 5′- CTAGCCCATCTCCCAAAGATCC -3′; and *Tlr5*-null (Exon4)-Rev 5′- AAACAGTGAGACAAAGCTCCCT -3′). Amplification was performed in a 10μl reaction volume containing 2.5 μl diluted DNA, 1× New England Biolabs (NEB) PCR buffer, 0.75mM MgCl_2_, 0.2mM dNTPs, 0.25μM each primer and 0.0375u Taq polymerase (NEB) for 30 cycles of 94°C for 30 sec, 60°C for 30 sec and 72°C for 30 sec. The wild-type allele produced a 350-bp product while the *Tlr5*-null allele produced a 144-bp product. All mice used in this study were on an inbred and retained MRL/*lpr* background. N1F1 heterozygotes were transferred to Virginia Tech. At Virginia Tech, mice were maintained in a specific pathogen-free animal facility. *Tlr5-null* mutant mice were backcrossed to produce N2F1 heterozygotes, which were intercrossed to produce experimental *Tlr5* ^+/+^, *Tlr5* ^+/-^ and *Tlr5* ^-/-^ MRL/*lpr* littermates. To validate our deletion approach, renal transcript levels of *Tlr5*, *Tlr7* and *Tlr9* were measured. Only *Tlr5* was deleted in the kidney of *Tlr5* ^-/-^ MRL/*lpr* mice (**Supplementary Figure 1**), suggesting that the observed disease phenotype with *Tlr5* deletion was not due to changes of two TLR genes known to affect lupus, *Tlr7* or *Tlr9*. All procedures were carried out according to an approved Institutional Animal Care and Use Committee protocol (No. 21-051). *Tlr5* ^+/+^, *Tlr5* ^+/-^ and *Tlr5* ^-/-^ MRL/*lpr* littermates (n=5, 7 and 7, respectively) were generated through heterozygous intercross, housed by sex and genotype after weaning, and continuously monitored every week for body weight and proteinuria till euthanasia at 15 weeks of age. All other phenotypic analyses were performed with samples collected upon euthanasia at 16 weeks of age. Fecal pellets were collected at 8 and 15 weeks of age. The analyses of intestinal permeability (n=4-5/group at 7 weeks of age) and host metabolism (n=4-5/group at 15 weeks of age) were each performed with littermates generated from a new round of heterozygous intercross.

### 2.2 Cell isolation

Total splenocytes were isolated with red blood cell exclusion following established methods (18, 19). For renal leukocyte isolation, a modified version of our previously reported protocol (20) was employed. Briefly, kidneys were finely minced into 1- to 2-mm^3^ pieces and digested in a 5 ml solution of digestion buffer containing 1 mg/ml collagenase and 0.2 mg/ml DNase I (Sigma‐Aldrich, St. Louis, MO) in RPMI 1640 medium supplemented with 10 mM HEPES, followed by a 1-hour incubation at 37°C with continuous gentle stirring. Subsequently, 10 ml of ice-cold phosphate buffered saline (PBS) with 10 mM EDTA was added and incubated for 10 minutes on ice. The resulting cell suspensions were filtered through a 70-µm strainer, washed with 10 ml of HBSS-full [HBSS without Ca^2+^ and Mg^2+^ (Life Technologies, Carlsbad, CA) containing 5 mM EDTA, 0.1% bovine serum albumin (BSA), and 10 mM HEPES], then centrifuged at 2000 rpm for 10 minutes at room temperature. The cell pellets were resuspended in 5 ml of 30% stock isotonic Percoll [SIP; 100% SIP prepared as 1 part volume of 10× PBS and 9 parts volume of Percoll (Fisher Scientific, Hampton, NH)]. These suspensions were gently loaded on a 37% (5 ml) – 70% (5 ml) SIP gradient and subsequently centrifuged for 30 minutes at 1000×*g* at room temperature with deacceleration set as 0. Enriched leukocytes were collected from the interface between 37% and 70% SIP. Splenocytes and renal leukocytes were then processed for flow cytometry analysis as described below.

### 2.3 Flow cytometry

Single-cell suspensions were initially blocked with an Fc receptor blocker, anti-mouse CD16/32 (Thermo Fisher Scientific, Waltham, MA), on ice for 10 minutes, then stained with fluorochrome-conjugated antibodies for 15 minutes in the dark in accordance with previously established protocols (18, 19). All flow cytometry analyses were conducted exclusively on the live cell populations, which was achieved by excluding dead cells through staining with Zombie Aqua (BioLegend, San Diego, CA). To quantify type 1 conventional dendritic cells (cDC1) and T helper-17 (Th17) cells, the following anti-mouse primary antibodies were utilized: CD45-APC/Cy7, CD11c-BV421, CD11b-AF700, MHCII-FITC, Ly6C-APC-Cy7, Ly6G-PE, CD3-FITC, CD4-APC, FOXP3-BV421, and RORγT-PE (BioLegend). Activated cDC1 cells were identified as CD45^+^ Ly6G^-^ MHCII^+^ CD11c^+^ CD11b^-^ CD86^+^. Th17 cells were identified as CD45^+^ CD3^+^ CD4^+^ RORγT^+^. Analysis was carried out using a BD FACSAria Fusion flow cytometer (BD Biosciences, San Jose, CA), and flow cytometry data were subsequently analyzed using the FlowJo software (FlowJo, Ashland, OR).

### 2.4 Renal function analyses

Fixed kidney tissues were embedded in paraffin, sectioned, and subjected to Periodic Acid-Schiff (PAS) staining at the Histopathology Laboratory, Virginia-Maryland College of Veterinary Medicine. Kidney histopathology was evaluated on a scale from 0 to 3 for various parameters, including glomerular nephritis components such as cellularity, mesangial matrix, necrosis, percentage of sclerotic glomeruli, and presence of crescents, as well as tubulointerstitial nephritis and perivascular infiltration. Slides were scored by a board-certified veterinary pathologist (T. Cecere) in a blinded fashion (21). Proteinuria levels were determined using a Pierce Coomassie Protein Assay Kit (Thermo Fisher Scientific).

### 2.5 Immunohistochemistry

Kidneys and spleens were embedded in Tissue-Tek OCT Compound (Sakura Finetek, Torrance, CA) and rapidly frozen in a dry ice and 2-methylbutane freezing bath. The frozen OCT-embedded samples were cryosectioned, and unstained slides were stored at -80°C. Subsequently, these frozen slides were allowed to reach room temperature and dry for 30 minutes before fixation in -20°C cold acetone for 10 minutes. After a wash in PBS, the slides were blocked with PBS containing 1% BSA and anti-mouse CD16/32 (1:100, BioLegend) for 40 minutes at room temperature. Following the blocking step, the slides were incubated with a mixture of fluorochrome-conjugated antibodies for 2 hours at room temperature in a humid box. Finally, the slides were mounted using Prolong Gold containing DAPI (Life Technologies). The immunohistochemical analysis utilized the following anti-mouse antibodies: complement C3-FITC (1:200, Cedarlane, Cat# 1850362A); IgG2a-PE (1:200, BioLegend, Cat# 407107); CD3-APC (1:40, BioLegend, Cat# 100235); GL7-AF488 (1:80, BioLegend, Cat# 144606); and IgD-PE (1:100, BioLegend, Cat# 405705). Slides were examined and imaged using a Zeiss LSM880 confocal microscope. Image processing and quantification of the fluorescent intensity was performed with ImageJ and ZEN 2.1 Lite software equipped with a 20× objective.

### 2.6 16S rRNA sequencing

Fecal pellets were collected weekly from each mouse directly from the anus to maintain sterile conditions and immediately stored at -80°C until processing. Subsequently, the samples were homogenized, cell lysed, and DNA was extracted using a phenol-chloroform method as previously described (16, 17, 22–24). PCR were performed and purified amplicons were sequenced bidirectionally on an Illumina MiSeq at Argonne National Laboratory. The sequencing data were deposited in the NCBI SRA database with BioProject number PRJNA1021666.

### 2.7 RT-qPCR

Spleen tissues was homogenized using a TissueLyser II homogenizer (Qiagen). Total RNA was extracted from the homogenized samples using the RNeasy Plus Universal Kit from Qiagen (Hilden, Germany) following the manufacturer’s instructions. Genomic DNA contamination was eliminated through digestion with RNase-free DNase I (Qiagen). Reverse transcription (RT) was conducted using the iScript cDNA Synthesis Kit from Bio-Rad (Hercules, CA). Quantitative PCR (qPCR) was performed with the iTaq Universal SYBR Green Supermix from Bio-Rad on an ABI 7500 Fast Real-Time PCR System from Applied Biosystems (Waltham, MA). Relative gene expression was calculated, with *18S* rRNA serving as the housekeeping gene for normalization. Triplicate reactions were run for each sample. Primer sequences are available upon request.

### 2.8 ELISA

Serum samples were obtained by separating serum from blood after allowing it to clot at room temperature for 2 hours, and the collected serum was subsequently stored at -80°C. Anti-double-stranded (ds)DNA IgG levels were quantified as previously described (25).

### 2.9 Intestinal permeability

*In vivo* intestinal permeability assay was conducted using 4-kDa FITC-conjugated dextran (Sigma-Aldrich). In brief, mice were subjected to six hours water deprivation period and subsequently administered FITC-dextran dissolved in PBS at a concentration of 40 mg/100 g body weight (approximately 300 μL/mouse) via oral gavage. After one hour, mice were euthanized, and blood was collected and kept in the dark until serum separation. Serum was then diluted at a 1:3 ratio with PBS and added to a 96-well microplate in duplicate. The FITC concentration was determined using GloMAX^®^ (Promega, Madison, WI) with excitation at 485 nm and emission at 528 nm, with serially diluted FITC-dextran as the standard for calibration.

### 2.10 Metabolic analyses

Body fat, lean mass and fluid percentage of the total body mass were assessed via nuclear magnetic resonance using an LF90 Bruker (Billerica, MA). Fatty acid oxidation was assessed using radiolabeled fatty acid ([1-^14^C]- palmitic acid, American Radiolabeled Chemicals, St. Louis, MO.) to quantify ^14^CO_2_ production and ^14^C-labeled acid-soluble metabolites. Samples were incubated in 0.5 μCi/mL of [1-^14^C]-palmitic acid for 1 hour after which the media was acidified with 200 μL 45% perchloric acid for 1 hour to liberate ^14^CO2. The ^14^CO2 was trapped in a tube containing 1 M NaOH, which was then placed into a scintillation vial containing 5 mL scintillation fluid. The vial’s ^14^C concentrations were measured on a 4500 Beckman Coulter scintillation counter. Acid soluble metabolites were determined by collected the acidified media and measuring ^14^C levels. Metabolic efficiency was expressed as a ratio of ^14^CO_2_ production (complete palmitate oxidation) to acid soluble metabolites (incomplete palmitate oxidation). Glucose oxidation was measured with methods similar to that of fatty acid oxidation with the exception of the substitution of radiolabeled [U-^14^C]-glucose. Total protein content in the tissue homogenates was measured via a bicinchoninic acid procedure (Thermo Fisher Scientific, Waltham, MA.) and oxidation values were normalized to total protein content.

### 2.11 Statistical analyses

Most comparisons involving three genotypes were analyzed with one-way ANOVA. Two-way ANOVA was employed for the proteinuria time course data analysis. Data are shown as average ± standard deviation (SD). Statistical significance was defined as *p*<0.05 (*p<0.05, **p<0.01, ***p<0.001, ****p<0.0001). All statistical analyses were carried out using GraphPad Prism software (Boston, MA).

## 3 Results

### 3.1 *Tlr5* deficiency deteriorates lupus nephritis by promoting renal leukocyte infiltration and deposition of complement C3 and IgG

Lupus nephritis affects up to 60% of SLE patients and is one of the most severe manifestations of lupus (26, 27). We had hypothesized that a leaky gut would contribute to SLE-like autoimmunity in lupus-prone MRL/*lpr* mice through bacterial flagellin-mediated activation of TLR5, and that global *Tlr5* deficiency would attenuate disease. Surprisingly, *Tlr5* deficiency exacerbated lupus nephritis in MRL/*lpr* females (**Figure 1**) but not MRL/*lpr* males (**Supplementary Figure 2**). From now on, we would focus on female mice as lupus has a strong female bias. MRL/*lpr* mice lacking *Tlr5* exhibited significantly exacerbated proteinuria early and before the proteinuria rose in either wild-type or heterozygous mice (**Figure 1A**). Notably, the level of proteinuria reached over 2,000 mg/dL in *Tlr5* ^-/-^ MRL/*lpr* mice, a level that had never been seen in our colony of MRL/*lpr* mice. In fact, we lost two *Tlr5*-deficient mice between 15 and 16 weeks of age (after the last urine collection) due to extremely high levels of proteinuria. This suggests that *Tlr5* deficiency may facilitate lupus-associated renal failure. Analysis of kidney histopathology (**Figure 1B**) showed that *Tlr5*-deficient mice had significantly higher pathological scores in tubular damage, hypercellularity and glomerulonephritis (**Figure 1C**; **Supplementary Figure 3**).

**Figure 1:** *Tlr5* deficiency deteriorates lupus nephritis. **(A)** Levels of proteinuria over time. n=5-7/group. **(B)** Representative PAS-stained kidney glomeruli. Bar equals 200 µm. **(C)** Histopathological scores showing tubular damage and hypercellularity, as well as accumulative glomerulonephritis scores. n=3-4/group.

Interferons, particularly type I interferons, play a central role in the pathogenesis of lupus (28). Thus, we measured the expression of interferon responsive genes (IRGs) in the kidney (**Supplementary Figure 4**) and found that the levels of *Cxcl1* and *Isg15* were upregulated in *Tlr5*-deficient MRL/*lpr* mice. Consistently, we found significantly increased renal infiltration of Th17 cells (**Figures 2A, B**) and activated cDC1 cells (**Figures 2C, D**) with *Tlr5* deficiency. No significant differences were observed among experimental groups in the other immune cell subsets (**Supplementary Figure 5**). Taken together, these findings indicate that *Tlr5* deficiency promotes IRG expression and facilitates Th17 and activated cDC1 cell infiltration into the kidney to deteriorate lupus nephritis.

**Figure 2:** *Tlr5* deficiency promotes renal leukocyte infiltration. **(A, B)** Representative FACS plots **(A)** and bar chart **(B)** showing the percentage of Th17 cells in the kidney. Plots were pre-gated on CD45^+^ CD3^+^ CD4^+^ cells. **(C, D)** Representative FACS plots **(C)** and bar chart **(D)** showing the percentage of CD86^+^ (activated) cDC1 cells in the kidney. Plots were pre-gated on CD45^+^ Ly6G^-^ MHCII^+^ CD11c^+^ CD11b^-^ cells. n=4-6/group.

The interplay among T cells, complement C3, and IgG immune complexes in the kidney is a central mechanism in the pathogenesis of lupus nephritis (29). We thus performed immunohistochemical analyses of renal deposition of complement C3 and IgG2a, the pathogenic IgG isotype, as well as the infiltration of CD3^+^ T cells. While the serum levels of anti-dsDNA IgG did not differ (**Supplementary Figure 6A**), renal deposition of C3 and IgG2a was noticeably higher for *Tlr5^-/-^* MRL/*lpr* mice compared to the wild-type and heterozygous littermate controls (**Figure 3A**). Quantification of the fluorescence intensity confirmed that they were indeed significantly higher (**Figure 3B**). Furthermore, increased intensity of CD3 fluorescence was observed in the kidney of *Tlr5*-deficient MRL/*lpr* mice (**Figure 3B**), indicating aggravated renal infiltration of T cells. These results suggest that *Tlr5* deficiency promotes renal deposition of C3 and IgG and facilitates T cell infiltration into the kidney to exacerbate lupus nephritis.

**Figure 3:** *Tlr5* deficiency exacerbates renal deposition of complement C3 and IgG and increases T cell infiltration. **(A)** Representative immunohistochemical images of kidney sections. Bar equals 100 μm. **(B)** Fluorescence intensity was quantitated using ImageJ. MFI values are shown. n=3-4/group.

### 3.2 *Tlr5* deficiency exacerbates lymphoproliferation by promoting germinal center reaction and suppressing regulatory lymphocytes

Female MRL/*lpr* mice lacking *Tlr5* exhibited significantly worse splenomegaly (**Figure 4A**) and lymphadenopathy (**Figures 4B, C**) than the wild-type littermates. These results suggest that *Tlr5* deficiency has an influence on lymphoproliferation in MRL/*lpr* mice. To elucidate the mechanism by which *Tlr5* deficiency exacerbates lymphoproliferation, we investigated the formation of germinal centers in the spleen. We observed significantly increased expression of GL7 on splenic sections compared to wild-type MRL/*lpr* mice (**Figures 5A, B**), indicating the promotion of germinal center reaction in *Tlr5*-deficient MRL/*lpr* mice. We also quantified splenic FOXP3^+^ regulatory T (Treg) cells (**Figure 5C**) and two types of regulatory B (Breg) cells, marginal zone B cells and transitional 2-marginal zone precursor B cells (**Figure 5D**). *Tlr5* deficiency significantly suppressed both Treg and Breg cells compared to the wild-type or heterozygous littermates. These findings indicate that *Tlr5* deficiency exacerbates lymphoproliferation in MRL/*lpr* mice by promoting germinal center reaction and suppressing regulatory lymphocytes in the spleen.

**Figure 4:** *Tlr5* deficiency exacerbates lymphoproliferation. **(A, C)** Splenomegaly **(A)** and lymphadenopathy (**B**, mesenteric; **C**, axillary and cervical) characterized by increased lymphoid organ-to-body weight ratios. n=4-6/group.

**Figure 5:** *Tlr5* deficiency promotes germinal center reaction and suppresses regulatory lymphocytes in the spleen. **(A)** Representative immunohistochemical images of splenic sections. Bar equals 100 μm. **(B)** Mean fluorescence intensity (MFI) of GL7 was quantitated using ImageJ. n=3/group. **(C)** Representative FACS plots (left) and bar chart (right) showing the percentage of regulatory T cells (Treg) cells in the spleen. Plots were pre-gated on CD3^+^ CD4^+^ cells. n=3-4/group. **(D)** Percentages of marginal zone B cells (MZB; CD19^+^ IL10^+^ CD21^+^ CD24^hi^ IgM^+^ CD23^-^) and transitional 2-marginal zone precursor B cells (T2-MZP; CD19^+^ IL10^+^ CD21^+^ CD24^hi^ IgM^+^ CD23^+^) in the spleen. n=4-5/group.

### 3.3 *Tlr5* deficiency induces dynamic changes in fecal microbiota but does not affect the existing leaky gut or host metabolism

Changes in the dynamics of microbiota have been shown to trigger autoimmunity (22, 30) or modify autoimmunity (31). *Tlr5* deficiency in mice of C57BL/6 (B6) background has been shown to induce significant alterations in the intestinal microbiota, leading to a complex interplay of effects including the development of metabolic syndrome and increased susceptibility to colitis (32, 33). To test if *Tlr5* deficiency affects the gut barrier in MRL/*lpr* mice, we gavaged the mice with FITC-dextran and found that there was no difference in small intestinal permeability with or without TLR5 (**Supplementary Figure 6B**). Next, we investigated whether the deficiency in *Tlr5* could implicate the gut microbiota in MRL/*lpr* mice. We analyzed the fecal microbiota with 16S rRNA sequencing and mapped the composition of the gut microbiota using β-diversity. Two mouse ages were analyzed, 8 (pre-disease stage; data not shown) and 15 weeks (late-disease stage), with only 15 weeks of age showing significant differences. Clear distinctions were found among the 15-week fecal microbiotas of *Tlr5*-deficient, heterozygous and wild-type MRL/*lpr* mice (**Figure 6A**). In addition, many significant changes were identified at different taxonomical levels. At the Class level, the relative abundances of Erysipelotrichia and Alphaproteobacteria/Gammaproteobacteria (combined) were significantly decreased, whereas Mollicutes and Deltaproteobacteria significantly increased, with *Tlr5* deficiency (**Figure 6B**). At the Order level, Desulfovibrionales were more abundant in the *Tlr5*-deficient mice whereas Bifidobacteriales were mostly removed from these mice (**Figure 6C**). At the Family level, *Lachnospiraceae*, *Intestinimonas*, *Oscillibacter* and *Ruminiclostridium* were more abundant in *Tlr5*-deficient mice, whereas *Romboutsia* were significantly lower in relative abundance with *Tlr5* deficiency (**Figure 6D**). Finally, increases of *Odoribacter*, *Allistipes*, *Rikenella*, and *Intestinimonas* were found at the Genus level in the *Tlr5*-deficient MRL/*lpr* mice compared to wild-type MRL/*lpr* littermates (**Figure 6E**). However, contrary to the observations in *Tlr5* ^-/-^ B6 mice (33), there was no change in host metabolism with or without *Tlr5* in MRL/*lpr* mice (**Supplementary Figure 7**). These results indicate that *Tlr5* deficiency induces dynamic changes in fecal microbiota but does not affect the existing leaky gut (23) or host metabolism in lupus-prone MRL/*lpr* mice.

**Figure 6:** *Tlr5* deficiency induces dynamic changes in fecal microbiota. **(A)** Unweighted UniFrac analyses with 3D plotting by principal component (PC) distances. **(B–D)** Relative abundance at Class, Order and Family levels, respectively. n=5-7/group.

## 4 Discussion

In this study, by creating global *Tlr5* deletion on the MRL/*lpr* background, we aimed to delineate the role of TLR5 in autoimmune lupus through a loss-of-function approach. We showed that *Tlr5* deficiency in MRL/*lpr* mice, instead of attenuating disease as we had hypothesized, exacerbated lupus. Mechanistically, the loss of TLR5 affected the spleen by promoting germinal center reaction and decreasing the frequencies of Treg and Breg cells. While we did not analyze the lymph nodes, it is reasonable to anticipate similar results, as both splenomegaly and lymphadenopathy are impacted by lymphoproliferation in the MRL/*lpr* mouse model. The loss of TLR5 also affected the kidney by promoting IRGs, increasing deposition of complement C3 and IgG, and facilitating the infiltration of T cells (particularly Th17 cells) and activated cDC1 cells. The collective functions of these changes led to aggravated glomerulonephritis with *Tlr5* deficiency. These results suggest that global *Tlr5* deletion exacerbates both lymphoproliferation and glomerulonephritis, two hallmarks of SLE-like disease in MRL/*lpr* mice.

It is known that *Tlr5*-deficient B6 mice are susceptible to intestinal proinflammatory gene expression elevation (34). However, the role of TLR5 in SLE and associated complications was unknown. Our findings from this study shed light on how *Tlr5* deficiency influences systemic and renal inflammation in the context of SLE. The observed impact of *Tlr5* deficiency on lymphoproliferation and the development of massive splenomegaly and lymphadenopathy underlying the significance of TLR5 in systemic immune homeostasis. Therefore, it appears that TLR5 can modulate immune responses beyond its basic function of recognizing bacterial flagellin (12). The enlargement of spleen and lymph nodes with *Tlr5* deficiency could be attributed to dysregulated immune activation, leading to lymphoid tissue accumulation of immune cells, exacerbation of autoimmune responses, and systemic inflammation that are characteristics of SLE. In addition, the promotion of germinal center B cells (GL7^+^) and the suppression of regulatory lymphocytes in *Tlr5*-deficient MRL/*lpr* mice highlight the intricate balance between effector and regulatory components of the immune system. The expansion of germinal center B cells suggests heightened antibody production and immune responses, which can contribute to autoantibody production in SLE (35). Concurrently, the suppression of regulatory lymphocytes may further tip the balance toward immune dysregulation, amplifying the autoimmune response (36). IRGs are often overexpressed in individuals with lupus (37), indicating a crucial role for interferon signaling in the pathogenesis of the disease. Our results showed that *Tlr5* deficiency upregulated the expression levels of *Cxcl1* and *Isg15*. CXCL1 has been found to be significantly upregulated in lupus (38) and the expression of ISG15 is elevated in SLE patients and correlates with disease activity (39). Notably, while both type 1 and type 2 interferons are elevated in human SLE (40), it appears that they have opposite functions in MRL/*lpr* mice. Type 1 interferons can be protective (41) whereas interferon-γ contributes to lupus-like disease in MRL/*lpr* mice (42). Our presented data cannot differentiate whether the induction of *Cxcl1* and *Isg15* is due to type 1 or type 2 interferon signaling. Nonetheless, our observations in *Tlr5* ^-/-^ MRL/*lpr* mice suggest exacerbated systemic inflammation with global deficiency of TLR5. Furthermore, our results indicate exacerbation of renal inflammation with *Tlr5* deficiency in MRL/*lpr* mice. The infiltration of inflammatory cells and immune complex deposition in renal tissues intensify local inflammation, ultimately contributing to kidney damage. Consistently, we observed aggravated glomerulonephritis with *Tlr5* deficiency. These results emphasize the role of TLR5 in modulating kidney-specific immune responses in SLE.

The gut microbiota is increasingly recognized as a critical player in the development and modulation of autoimmune diseases, including SLE (43) and graft-versus-host disease, which shares some clinical signs as SLE (44, 45). Our observation of distinct differences in the fecal microbiota diversity among *Tlr5-*deficient, heterozygous, and wild-type MRL/*lpr* mice underscores a role of TLR5 in shaping the gut microbiota. *Tlr5* deficiency can alter the recognition and response to specific microbial components, leading to changes in the microbial community (46). These alterations are particularly relevant in the context of autoimmunity, as changes in microbiota composition are known to influence immune responses against self (5). One noteworthy finding is the decrease in Erysipelotrichia and the increase in Mollicutes at the Class level in *Tlr5*-deficient MRL/*lpr* mice compared to their wild-type littermates. These changes may indicate a shift in the relative abundance of specific bacterial taxa that could influence the immune balance in the gut. Specifically, increased Mollicutes has been associated with SLE (47). Alterations were also observed in the Order-level composition, including the increase in Desulfovibrionales and partial removal of Bifidobacteriales. Desulfovibrionales are sulfate-reducing bacteria that are part of the normal gut microbiota, but their increased levels may contribute to colitis development (48). Bifidobacteria, on the other hand, are beneficial bacteria; and reduced abundance of Bifidobacteriales in the gut microbiota has been associated with atopic disease (49). Therefore, the shift from Bifidobacteriales to Desulfovibrionales with *Tlr5* deficiency is consistent with the heightened inflammation observed in these mice. At lower taxonomic levels, several differences in the abundance of specific bacterial families and genera are commendable. The increased abundance of *Lachnospiraceae*, *Intestinimonas*, *Oscillibacter*, and *Ruminiclostridium* in *Tlr5*-deficient MRL/*lpr* mice may have functional implications, as these bacteria can produce metabolites that influence host immune responses (50–54). We have previously reported that *Lachnospiraceae* is increased in the MRL/*lpr* mouse model (22). *Oscillibacter*, on the other hand, is increased in autoimmune polyendocrine syndrome type 1 (APS-1) (55). Additionally, the increases in genera such as *Odoribacter*, *Allistipes*, *Rikenella*, and *Intestinimonas* suggest a potential shift in the microbial community toward taxa that may contribute to immune dysregulation (54, 56–58).

Interestingly, we observed that *Tlr5* deficiency had a minimal effect, if any, on male MRL/*lpr* mice. We have previously shown that the effect of gut microbiota in male MRL/*lpr* mice is suppressed by hormones, as castration allowed for the changes of microbiota to modulate disease (23). Since we hypothesize that changes of gut microbiota could be a mechanism for disease exacerbation in *Tlr5*-deficient MRL/*lpr* mice, we also postulate that this mechanism is suppressed in male mice.

In conclusion, this study provides valuable insights into the multifaceted impact of TLR5 on immune responses in the context of SLE. These findings underscore the complex interplay between innate immunity, adaptive immune responses, and tissue-specific inflammation in autoimmune diseases. In addition, our study provides evidence that *Tlr5* deficiency in MRL/*lpr* mice is associated with changes of the gut microbiota composition. These changes may be consequences of the immune dysregulation, which can, in turn, influence the development and progression of SLE-like disease. Future research into the molecular mechanisms underlying these observations is essential for a comprehensive understanding of SLE pathogenesis and for the development of targeted therapeutic interventions against the autoimmune disease.

## Data availability statement

The data presented in the study are deposited in the NCBI SRA repository, accession number PRJNA1021666.

## Ethics statement

The animal study was approved by Virginia Tech Institutional Animal Care and Use Committee. The study was conducted in accordance with the local legislation and institutional requirements.

## Author contributions

RA: Writing – original draft, Writing – review & editing. DO: Writing – review & editing. RE: Writing – review & editing. AS: Writing – review & editing. RL: Writing – review & editing. MA: Writing – review & editing. SS: Writing – review & editing. JN: Writing – review & editing. SK: Writing – original draft. TC: Writing – review & editing. RM: Writing – original draft. CR: Writing – review & editing. XL: Writing – original draft, Writing – review & editing.
